The article "Landscape Fusion Method Based on Augmented Reality and Multiview Reconstruction" was published in 2022. Journal: Appl Bionics Biomech.

# Landscape Fusion Method Based on Augmented Reality and Multiview Reconstruction

**DOI:** 10.1155/2022/5894236

**Published:** 2022-07-29

**Authors:** Genlong Song, Yi Li, Lu-Ming Zhang

**Affiliations:** ^1^College of Computer Science and Artificial Intelligence, Wenzhou University, Wenzhou, Zhejiang, China; ^2^Key Laboratory of Crop Harvesting Equipment Technology of Zhejiang Province, Jinhua Polytechnic, Jinhua, Zhejiang, China

## Abstract

This paper proposes a fused landscape augmented reality method based on 3D model multiview reconstruction. Based on the principles related to augmented reality technology, the proposed method uses natural features of images for training and extraction, which solves the problems of convenience and aesthetics caused by artificial signs. By extracting and training natural features at different scales of the acquired images, Harris and FREAK algorithms are used to extract features and create binary descriptors for real-time acquired images. Feature matching is performed on the above two features to estimate the location where the reconstructed model will appear. At the same time, for the difficulties of 3D model reconstruction requiring relevant expertise and the defects of poor reconstruction effect, the SFM algorithm is used for multiview reconstruction of landscape models to realize the augmented reality fusion method of natural scenes and landscape models. After the experiments, the fusion achieved by this method works well, which proves that the method is feasible and has potential.

## 1. Introduction

More and more phenomena are showing that human activities are constantly damaging the natural world, and the survival of the landscape is facing big problems. Moreover, due to the single presentation form of landscapes in natural scenes, people have gradually lacked the freshness of these landscapes. Therefore, how to protect landscapes effectively in natural scenes and develop distinctive landscape presentation forms has become a research hotspot in recent years. The emergence of virtual reality [1] has brought many researchers a new sense of vision. Virtual reality abstracts the user from their surroundings and presents them with visual and auditory stimuli, which allows them to find a different feeling in completely different environment [2, 3]. Although virtual reality has a strong sense of immersion, the user experience cost is high due to the expensive and difficult to carry equipment for realizing virtual reality, and after a long time of use, it will cause dizziness, and the lasting comfort experience is insufficient, so virtual reality has market development limitations for a long time. Based on this, the field of research in augmented reality emerged.

Augmented reality (AR) [4] is a further development of virtual reality, which combines real-world scenes with virtual visual interaction and enhances the real world by applying models, sounds, lights, etc. In recent years, due to the emergence of the new crown epidemic, people's travel has been greatly restricted, and people's appreciation of the unique beauty of various landscapes in natural scenes is inhibited. AR technology has created a new way for people to contact the outside world. Through research [5], it was found that, during the pandemic, digital technologies such as AR have played a major role in people's need to help fight the pandemic. From the term “augmented reality” proposed [6] to the present, from a single limited application scenario at the beginning to a wide range of applications in medical [7], cultural [8], education [9], tourism [10], entertainment [11], and social interaction [12], AR has proven its huge development potential.

The design of various landscapes in natural scenes plays a vital role in the development of people's physical and mental health, especially the design of green landscapes [13]. The epidemic has inhibited people's freedom of travel and hindered people from feeling the meaning of the landscape in the outside world. Using AR technology, people can feel the unique expression of the outdoor landscape indoors and present it in the form of a realistic model, leaving people with an alternative charm of the corresponding landscape. It reduces the regret that people cannot visit the scene of the landscape in person due to the epidemic and economic reasons and cannot truly experience the natural scene landscape and satisfies the arbitrariness of people's appreciation of the landscape.

In response to the development limitations of AR technology in natural scenes, we combined the implementation of AR technology and the characteristics of landscape in natural scenes to realize an AR fusion method, which includes AR creation, multiview reconstruction of landscape models, and virtual-real synthesis presentation.

In this integrated method, people can enjoy the sights of different landscapes. By rotating the identification map or camera equipment, they can view the state of various perspectives of the landscape in all directions. Because we use the multiview reconstruction technology of the model to reconstruct the model of the real-world landscape, it is more realistic than the model reconstruction through 3D model software and can display the characteristic image of the landscape in the natural scene to the greatest extent. This multimedia fusion method based on AR technology only needs one camera device and one display device, with relatively low cost and simple operation mode, which greatly satisfies the general public's desire for AR technology.

In this paper, we propose an augmented reality method of fused landscape combined with 3D model multiview reconstruction based on the implementation principle of augmented reality technology. By training and extracting the natural features of images, we solve the problems of convenience and aesthetics caused by artificial marking features. At the same time, the method uses the method of Harris corner point detection for feature extraction of the video frame images captured in real time. The FREAK algorithm is used to create binary feature descriptors for feature matching with images of natural scene landscapes from different angles that have completed feature training. Then, in combination with the projection matrix of the camera, the position of the virtual model rendering is calculated. The SFM algorithm is used for multiview reconstruction of landscape models to address the difficulties of 3D model reconstruction requiring relevant expertise and the shortcomings of poor reconstruction results. Finally, the reconstructed model is adjusted accordingly and then rendered on the location estimated by the above work through OpenGL to realize the augmented reality fusion method of natural scene and landscape model.

The rest of this article is organized as follows.  Section 2 describes some related works. Details about the implementation of this AR technique, such as feature training of images, and the work on multiview reconstruction of 3D models will be presented in Section 3. A demonstration about the results of this fusion method will be presented in Section 4. We will analyze the results and discuss the next direction of work in Section 5.

## 2. Related Work

Augmented reality (AR) technology provides a facility to overlay real scene flow images with virtual computer model images and allows viewers to observe the invisible heights of landscape architecture, which realistically represents alternative landscape changes [14, 15]. In recent years, digital technologies such as AR have been well developed in landscape architectural rendering.

This article [16] improved the modeling method of virtual reality technology, solved the shortcomings of low automation and weak applicability, and enhanced the application of virtual reality technology in interior landscape design. The paper [17] combined virtual reality and image processing technology to design an interactive architectural landscape roaming method, which solved the problems of low resolution and single system structure of the traditional landscape planning effect simulation system.

Rodrigues et al. [18] analyzed the possible benefits and limitations of traditional procedural modeling techniques applied to virtual heritage and proposed a complete methodology for the reconstruction of generated house models. In [19], Tobiáš et al. combined GIS technology, 3D software, and procedural modeling tools to present a landscape visualization model with a Czech castle and scenes around the castle, which allowed the user to easily identify from it historical landscape features and their changes over time. Zhou et al. [20] proposed an improved 3D reconstruction method by using a combination of point and line features. By integrating the extracted 3D lines into an optimized dense point cloud, the edges of landscape buildings were thus accurately reconstructed, and the accuracy, completeness, and efficiency of the reconstructed models were improved.

Yang et al. [21] proposed an interactive system based on 3D reconstruction method and AR. The system combined the reconstructed model with AR environment and provided a more convenient way to design and manage AR applications for building design. Tian et al. [22] proposed an effective AR occlusion processing method based on 3D reconstruction, which can determine whether there is occlusion between the real scene and the virtual model and process it in real time. This method greatly improved the practicality of AR systems.

A registration algorithm for an outdoor wearable AR system [23] improved registration accuracy by tracking natural features of outdoor scenes, which were captured by head-mounted displays. A realistic visualization method based on GIS was proposed by Ghadirian and Bishop [15], which dynamically enhanced the landscape view with the temporal changes of the modeling. By combining GIS and AR, the method showed the complex information of the landscape state and its dynamic changes in the natural scene. Portalés et al. [24] proposed the synergy between traditional close-range photogrammetry and AR. It visually constructed a hybrid urban space that users can walk through on-site, which created an AR environment that was physically impossible. The augmented reality-based 3D model visualization system [25] enabled users to easily feel the information of cultural landscapes in natural scenes outdoors. ARGIS system [26] was an outdoor registration mechanism of AR system that combined 3D GIS and AR system, which was much faster than visual tracking registration method. Combining traditional and indirect AR, Gimeno et al. [27] proposed a new mobile AR-based application to solve the problem of uncomfortable viewing caused by crowded crowds in museums, which allowed users to freely observe the enhanced museum environment without worrying about being blocked by other users. Kyriakou and Hermon [28] combined natural interaction with augmented reality and applied it in cultural heritage museums to solve the problem that cultural landscape and artifacts cannot be viewed or interacted. Ou et al. [29] combined deep learning with augmented reality and proposed a method to build a more efficient and restored landscape sandbox system with higher reproducibility and three-dimensional effect, made up for the shortcomings of the traditional landscape sandbox system. Allal-Chérif [30] analyzed the smart experience of using AR technology to bring tourists to visit the cathedral, which allowed them to easily see some places that were not open to the public due to the damage of cultural heritage landscape and helped tourists to understand the corresponding historical and cultural information.

The emergence of the above related works has facilitated the integration and interaction of AR technology and the model reconstruction techniques in natural scenes. However, it still has drawbacks, such as only applicable to indoor and large computational volume, the need to carry bulky equipment as well as the use of manual signs affects the convenience and aesthetics, and the authenticity of the presented landscape model is insufficient. The augmented reality fusion method proposed in this paper takes the natural features as the logo and uses AR technology and the multiview reconstruction method of the landscape model in the natural scene, which can show the realism of the virtual model in the augmented environment to the maximum extent.

## 3. Process

Augmented reality (AR) technology enhances the environment by mixing real world and virtual model. Milgram and Milgram et al. proposed a reality-virtual continuum [31, 32], which took the real and the virtual environment as two ends of the continuum. The middle part of them was called “mixed reality,” where the augmented reality was close to the real environment, and the augmented virtual was close to the virtual environment. Azuma [33] first proposed a scientific definition of augmented reality and pointed out that AR technology had three issues: (1) combination of virtual model and real world, (2) real-time interaction, and (3) 3D registration.

The implementation of this augmented reality fusion method requires the acquisition of natural scene video frames, as well as the feature recognition extraction of the captured video frame images in real time. The 3D registration technique is used to match the features of the acquired image with the template image and calculate the model view matrix. The model generated by the reconstruction of the scene landscape is rendered in the real scene through the virtual-real synthesis technology and finally presented on the display device, as shown in Figure 1.

### 3.1. Image Feature Training

Image feature training is an essential step in AR system. The feature training of the template image will have a crucial impact on the feature matching operation that follows. We will train the features at different resolutions, different angles, and different brightnesses.

Feature training is inseparable from the acquisition of image data, and the image acquisition needs to pay attention to the following points.

1. Perspective. Different angle changes will alter the visible area in the camera
2. Distance. The distance of the natural scene from the camera will change the resolution size of the subject for which the image features are to be trained
3. Illumination. Different lighting will change the brightness of the captured image. The local area brightness may be too high or too low
4. Shelter. Shelter will cause the captured image subject to be incomplete and affect the feature training effect

All of the above points will lead to changes in the number of captured image features, which may cause the later feature matching operations to fail and affect the implementation of the AR system.

In order to achieve more effective AR system for natural scenes and landscapes, image acquisition with different angles, resolutions, and illumination and presence of partial occlusion was performed for the set feature training targets. Some of the image acquisitions (take the example of partial image acquisition from different angles) are shown in Figure 2.

Here, the collected image data are trained for feature extraction by constructing DoG (difference of Gaussians) scale space. The DoG algorithm [34] is an algorithm for enhancing grayscale image and extracting feature point. By using the following Gaussian kernel functions with different parameter *σ* values for the acquisition images,

(1) $$\begin{array}{c} G\left(x,y,\sigma \right)=\frac{1}{\sqrt{2{\pi \sigma }^{2}}}e^{-\left(x^{2}+y^{2}\right)/2\sigma^{2}}, \end{array}$$

(2) $$\begin{array}{c} C\left(x,y,\sigma \right)=G\left(x,y,\sigma \right)*I\left(x,y\right), \end{array}$$

the convolution operation achieves the scale processing of the acquired image, i.e., the blurring degree of the image, where *G*(*x*, *y*, *σ*) is the Gaussian kernel function, (*x*, *y*) represents the image pixel position, *σ* is the scale factor, which determines the blurring degree of the image, ∗ is the convolution operation, *I*(*x*, *y*) is the input image, and *C*(*x*, *y*, *σ*) is the scale image under the corresponding *σ* value processing. Then, the two adjacent scale spaces of the image are differenced by

(3) $$\begin{array}{c} G=G\left(\sigma_{1}\right)-G\left(\sigma_{2}\right)=\frac{1}{\sqrt{2\pi }}\left(\frac{1}{\sigma_{1}}e^{-\left(x^{2}+y^{2}\right)/2\sigma_{1}^{2}}-\frac{1}{\sigma_{2}}e^{-\left(x^{2}+y^{2}\right)/2\sigma_{2}^{2}}\right), \end{array}$$

(4) $$\begin{array}{c} \text{DoG}=G*I\left(x,y\right), \end{array}$$

at the same size to obtain the DoG image, i.e., the Gaussian differential scale space. By using this method to train the image for feature extraction, many detailed features can be retained.

Image pyramids are downsampling the image to achieve the effect of image size transformation. A Gaussian image pyramid is formed by combining the Gaussian kernel function with the image pyramid. The results of the training (with some images trained at different angles as an example) are shown in Figure 3. In the training process, we set the minimum and maximum resolutions to 20 and 96, respectively, to construct the Gaussian differential scale space, and set the default image feature extraction degree values and initialization values. Based on the constructed scale space and image pyramids, we can obtain images of different resolutions. After the feature extraction training, the effect can be obtained as in Figure 4 (Taking the first set of images with different angles as an example, in order to compare the display effect of feature point extraction, we adjust the images of different sizes to the same size for display), where the green dots represent the feature points used for initial tracking and recognition of the image, the red boxes represent the features used for continuous tracking, and the blue numbers indicate the number of features for continuous tracking.

According to the trend of the number of feature points presented in Figure 4 (see Table 1 for the corresponding number of feature points and Figure 5 for the trend of the number of feature points), it can be concluded that the number of feature points extracted from the image has a significant trend of increasing as the image resolution rises. We divide multiple images of different resolutions for training to better realize an AR fusion system for natural scene landscapes.

### 3.2. 3D Registration

The augmented reality system superimposes the virtual three-dimensional model on the real scene, and the position of the superimposition in the real scene determines the final sense of reality. The 3D registration is the key step in the AR system that determines where the virtual model is presented in the real scene. Currently, 3D registration techniques can be divided into three categories: sensor-based, based on sensors and vision, and vision-based 3D registration techniques. Here, we use a 3D registration technique based on natural features in vision.

Natural features represent the information of the image, such as color, contour, edge gradient, and texture. A good natural feature should have the following characteristics: distinguishing: this feature point is distinguished from other feature points and thus is not easily identified by mistake; reliability: when the image is scaled, rotated, etc., the feature point can still be well recognized; and irrelevance: the image information contained in this feature should be independent of other feature points, so as to avoid data redundancy and increase computational complexity.

According to different feature extraction methods, natural features are divided into point, line, surface, texture, color, and statistical features. Point features are the most commonly used features in point-line-surface features. It is the basic feature of images and belongs to local features, such as corner and edge points. Corner points are one of the most typical feature points. Commonly used extraction methods for corners include curvature-based, gray-based, and edge-based extraction. Here is the corner feature extraction method based on grayscale change, Harris corner detection method.

Harris corner detection method [35] is a first-order derivative matrix detection method based on grayscale change, which has the characteristics of rotation invariance. It detects the local self-similarity of the image. That is, if its grayscale changes greatly when moving the feature window in the local area of the image, it is a corner point. Harris converts images in RGB format to grayscale images. Use formula (5) to calculate the grayscale change of the image *G*(*x*, *y*) after the point (*x*, *y*) is moved by (*α*,*β*).

(5) $$\begin{array}{c} V\left(x_{i},y_{i},\alpha ,\beta \right)=\underset{\left(x_{i},y_{i}\right)\in T\left(x,y\right)}{\sum }w\left(x_{i},y_{i}\right){\left[G\left(x_{i}+\alpha ,y_{i}+\beta \right)-G\left(x_{i},y_{i}\right)\right]}^{2}. \end{array}$$

*T*(*x*, *y*) is the image window centered at (*x*, *y*). (*x*_*i*_, *y*_*i*_) represents a point in the image window. *w*(*x*_*i*_, *y*_*i*_) represents the weighting function of the image at point (*x*_*i*_, *y*_*i*_). *G*(*x*_*i*_ + *α*, *y*_*i*_ + *β*) is the shifted image gray value, and *G*(*x*_*i*_, *y*_*i*_) is the original image gray value. According to the Taylor expansion method and the knowledge of the partial derivative function, the above formula is simplified to

(6) $$\begin{array}{c} V\left(\alpha ,\beta \right)≅\left[\alpha \;\beta \right]M\left[\begin{array}{c} \alpha \\ \beta \end{array}\right], \end{array}$$

where

(7) $$\begin{array}{c} M=\underset{\left(x_{i},y_{i}\right)}{\sum }w\left(x_{i},y_{i}\right)\left[\begin{array}{cc} G_{x_{\text{i}}}^{2} & G_{x_{i}}G_{y_{i}}\\ G_{x_{i}}G_{y_{i}} & G_{y_{\text{i}}}^{2} \end{array}\right]. \end{array}$$

According to the above formula, the points in the image are classified by calculating the corner response value *R*. The formula for calculating *R* is

(8) $$\begin{array}{c} R=\det M-c{\left(\text{trace}M\right)}^{2}. \end{array}$$

Here det*M* = *λ*_1_*λ*_2_, and trace*M* = *λ*_1_ + *λ*_2_, where *λ*_1_ and *λ*_2_ are the eigenvalues of the matrix *M*. *c* is an empirical constant. When the value range is [0.04, 0.06], the calculated corner response value *R* is the best, which is most suitable for corner detection. Thresholding is performed on the calculated corner response value *R*. When the value of *R* is greater than the threshold and is the local maximum value in the field of the point, the point is regarded as a corner point. After corner points are detected by the Harris corner point detection method, feature point descriptors are created for each corner point using the FREAK algorithm.

The FREAK (fast retina keypoint) algorithm [36] is an algorithm that detects key feature points based on the principle of object recognition by the human retina. Combined with the region division of the human retina for processing image information of different precision, the FREAK algorithm uses the most central point in the sampling structure as the feature point and the other circle centers as the sampling points. Since the FREAK algorithm uses a binary string to describe the feature points, it is expressed in Equation (9) as

(9) $$\begin{array}{c} F=\underset{0\leq a<N}{\sum }2^{a}T\left(P_{a}\right), \end{array}$$

where *P*_*a*_ denotes the sampled point pair and *N* denotes the length of the binary string used to describe the feature points, and the value of *T*(*P*_*a*_) is determined by formula (10), as follows.

(10) $$\begin{array}{c} T\left(P_{a}\right)=\left\{\begin{array}{c} 1,\text{if}\left(I\left(P_{a}^{r_{1}}\right)>I\left(P_{a}^{r_{2}}\right)\right),\\ 0,\text{otherwise}. \end{array}\right. \end{array}$$

Here, *I*(*P*_*a*_^*r*_1_^) and *I*(*P*_*a*_^*r*_2_^) denote the pixel values after Gaussian blurring of the previous and next sample points in sample point pair *P*_*a*_.

In order to create better feature descriptors, the FREAK algorithm filters the *N*-bit binary string to remove the nondiscriminatory descriptors and builds the matrix used to represent the binary descriptors. Each row of this matrix represents a binary descriptor of a feature point, and according to the sampling pattern of FREAK, there are 43 sampling points, so there is a *C*_43_^2^ = 903 sampling point pair; i.e., this matrix has 903 columns. Since the matrix is in binary, it is best to solve for the mean of the columns of the matrix with the mean at around 0.5. After that, all columns of the matrix are sorted according to their mean values, and the column closest to 0.5 is ranked first, and so on. The final number of columns of the most suitable binary descriptor is selected, i.e., the number of bits of the binary descriptor.

The formula

(11) $$\begin{array}{c} G=\frac{1}{M}\underset{P\in S}{\sum }\left(I\left(P^{r_{1}}\right)-I\left(P^{r_{2}}\right)\right)\frac{P^{r_{1}}-P^{r_{2}}}{\left\|P^{r_{1}}-P^{r_{2}}\right\|}, \end{array}$$

is used to calculate the gradient information of the sampled points, which is used to provide directions for the feature points. It guarantees rotational invariance, where *G* denotes local gradient information, *M* denotes the number of sampled point pairs, *S* denotes the set of sampled point pairs, and *P*^*r*_1_^ and *P*^*r*_2_^ denote the positions of the previous and next sample points in the sample point pair *P*. Since the FREAK descriptor has scale invariance and the Gaussian fuzzy makes the taken feature points have noise immunity and light invariance, the binary descriptor obtained by the FREAK algorithm to describe the feature points can be used for feature matching.

Finally, feature point matching is performed by the iterative closest point (ICP) algorithm. From there, the model view matrix, i.e., the rotation translation matrix, is calculated and combined with the camera projection matrix to estimate where the reconstructed model will appear in the real scene and complete the 3D registration.

### 3.3. Three-Dimensional Multiview Reconstruction

3D reconstruction is the process of reconstructing 3D information by using a single view or multiple views in the field of computer vision. Currently, 3D reconstruction mainly bases on monocular, binocular vision, and RGBD. For monocular vision, two main reconstruction categories exist: offline and online. The most classic of offline reconstruction is the SFM algorithm.

SFM (structure from motion) algorithm is an offline algorithm for 3D reconstruction based on disordered images with multiple views. Because the large numbers of images were required for reconstruction and the disorder between image data, various SFM strategies, such as incremental, hierarchical, and global, have emerged to efficiently process these image data for fast and accurate reconstruction. The incremental SFM algorithm [37] with strong robustness is the most frequently used. It first aligns two image data initially and then keeps adding one image to align and triangulate with the previous result. The overall reconstruction process of the incremental SFM algorithm is shown in Figure 6.

Before the SFM algorithm performs 3D reconstruction, some image processing work is performed. First, feature extraction algorithms such as SIFT are used to extract features from the input images. Feature matching is performed by calculating the correspondence between image feature points and selecting the set of feature point pairs that meet the requirements. Based on the matched feature point pairs, the geometric position of the camera and the feature matrix are estimated and optimized, and the matched feature point pairs are filtered and improved by the RANSAC algorithm: eight pairs of matching points are randomly selected from the matched pairs of feature points, and the basis matrix is solved. Then, the distance between the epipolar points and the epipolar line mapped by the basis matrix will be calculated. If the distance is less than the specified threshold, it is considered as an inner point. The number of inner points is counted and iterated by this, and the base matrix with the largest number of inner points is selected as the filtering result, and the matched point pairs that do not satisfy this base matrix are eliminated.

To carry out the reconstruction process, the SFM first selects two images for the initialized model reconstruction. The essential matrix is estimated from the positional information of one image and the matching point pair relationship with another image. Then, the matrix is decomposed to obtain the positional information of the other image. Afterwards, the alignment image is performed, and the set of feature points of the 2D image is transformed into the set of point clouds presented in 3D space by using triangulation to generate 3D spatial points. On this basis, the camera pose and feature points are optimally adjusted by using bundle adjustment to filter the points in 3D space that do not meet the requirements. After that, new image data are continuously added, and the above process is performed with the previous results until there is no suitable image data. Finally, the texture information is added to the obtained model mesh to present a more realistic 3D model. The effect is shown in Figure 7.

After the reconstruction, the model may be too large, and there are some poor reconstruction results. In order to facilitate the augmented reality fusion method to achieve better results, we can choose to use MeshLab tools or Autodesk Maya and other 3D modeling software to adjust the modeling results accordingly. The model will be resized to a suitable size and cropped of unwanted or bad effects from the reconstruction process. This operation makes the final model effect closer to the landscape rendering effect in the real scene and realizes the augmented reality fusion method of natural scene landscape.

### 3.4. Fusion of Virtual Model and Real World

The technology combines virtual model and real world by placing virtual objects in a real natural scene environment. Virtual objects in this context usually refer to virtual 3D models. Therefore, the reconstructed model largely influences the effect presented by the integration of the virtual model with the real world and determines the realism of the AR system. In this integration method, we use the 3D model files from the multiview reconstruction completed in the previous section to fuse with the natural scene.

Before rendering the reconstructed model by using OpenGL, the live image captured by the camera is called and displayed as a background through the cache. The perspective projection matrix is derived from the internal camera parameters and combined with the model view matrix calculated in the 3D registration section, i.e., the rotation translation matrix (R&T matrix), to estimate the position of the reconstructed model to be rendered in the background scene. Then, we proceeded to the rendering of the model. Since the model files we use contain information such as vertices, normals, textures, and materials, OpenGL is required to first read this information and render the corresponding mesh model. Then, rendering settings such as textures and lighting are performed to bring these together into the form of the model we need to present on the display device. Eventually, the background scene is combined with the rendered model to achieve the integration of the virtual model with the real scene. The fusion effect is shown in Figure 8.

## 4. Results

We use the ARToolKit framework under window10 system and Visual Studio2013 development tool for the realization of augmented reality fusion method. The equipment used here consists of a computer configured with an Intel(R) i7-8700 K@3.70 GHz CPU, 32 GB RAM, NVIDIA GeForce GTX 1080Ti graphics card, windows 11 OS, and a HD Pro Webcam C920 USB camera. The feature extraction of natural scene landscape is performed by training. Multiview model reconstruction is performed by using incremental SFM algorithm. The augmented reality fusion method of natural scene landscape is realized by combining 3D registration and virtual-real synthesis techniques, as shown in Figure 9.

We rotate the recognition image to present the effect image with different angles, as shown in Figure 10. The quantitative information of vertices, edges, and faces contained in the corresponding reconstructed model (the adjusted model) is shown in Table 2. At the same time, we can consider changing the size of the fusion model to better observe the presented natural scene landscape, as shown in Figure 11.

With the effect presented in Figures 9 and 10 and the quantitative information on vertices, edges, and faces contained in Table 2, we can see that the more complex the reconstructed model is, the more vertices, edges, and faces it contain, the relatively better the model reconstruction effect will be, and the more realistic the effect of fusion presented after combining with natural scenes.

According to the above effect video stream, we can get the corresponding frame rate from it as shown in Table 3. Calculating their average frame rates, we can obtain an average frame rate of 29.95 frames per second for scene 1, 29.975 frames per second for scene 2, and 30.1 frames per second for scene 3. Combined with the trend of frame rate variation (shown in Figure 12), we can find that the frame rate value always varies around 30 frames per second, with a maximum variation difference of 0.6 frames per second, which tends to be stable. It is concluded that the augmented reality fusion method of this natural scene landscape still has good stability and obvious effect in the case of large multiview reconstruction model.

## 5. Conclusion

This paper presents an augmented reality fusion method based on natural scene landscapes. The development of AR technology provides new ways of presenting natural scenic landscapes, and the emergence of the epidemic in recent years has allowed technologies such as AR to develop even more rapidly. The digitization of natural scenes and landscapes is usually presented in the form of pictures or videos, which are two-dimensional and lack realism. Over the years, people have long lost the novelty of this. Some of the applications have emerged on the combination of AR technology and natural scene landscape. However, the natural scene landscape model, especially the establishment of large landscapes, often requires modelers with professional backgrounds for model reconstruction, which is difficult to achieve, and the model differs significantly from the real landscape. To address these problems, we combine AR technology with multiview reconstruction of natural scene landscape to realize an augmented reality fusion method. Through this integrated method, people can enjoy a realistic representation of the outdoor landscape indoors. The results of the study prove that this method allows users to view different views of the landscape from different angles, which compensates for the fact that part of the landscape cannot be viewed from all sides. More importantly, the introduction of digital technology combined with the experience of realism further plays a role in preserving the natural scenic landscape.

However, this fusion method still faces some problems, such as the reconstructed model is too large to facilitate the implementation of augmented reality fusion method of multiobjective natural scenes and landscapes, as well as a single way of interaction, etc. Therefore, in future research activities, we will further improve the size of the reconstructed model while designing many different interaction methods to gradually realize a user-centered augmented reality fusion method with multiobjective natural field landscapes.

## Figures and Tables

**Figure 1:** Augmented reality fusion method implementation process.

**Figure 2:** Partial image acquisition data from different angles (the rotation angle from left to right in order is 0°, 45°, 90°, 135°, 180°, 225°, 270°, and 315°).

**Figure 3:** Feature point map of different angle images (the rotation angle from left to right in order is: 0°, 45°, 90°, 135°, 180°, 225°, 270°, and 315°).

**Figure 4:** Feature point diagrams at different resolutions (from left to right, the resolutions are (in DPI) 96.000000, 80.000008, 63.496048, 50.396847, 40.000004, 31.748022, 25.198421, and 20.000000).

**Figure 5:** Trend graph of the number of feature points (fset: the number of feature points used for continuous tracking; fset3: the number of feature points used for initializing tracking and recognizing images).

**Figure 6:** Incremental SFM algorithm reconstruction process.

**Figure 7:** The reconstructed effect of model.

**Figure 8:** Fusion effect.

**Figure 9:** AR fusion effect.

**Figure 10:** Different angle fusion effect.

**Figure 11:** The effect of the change in size of the fused model.

**Figure 12:** Frame rate trend graph.

**Table 1:** Number of feature points with different resolutions in different angle images.

	0°		45°		90°		135°	
Resolution	fset	fset3	fset	fset3	fset	fset3	fset	fset3
96.000000	476	651	407	637	337	640	392	688
80.000008	376	632	321	628	261	656	289	676
63.496048	254	595	214	592	180	647	180	635
50.396847	163	560	136	560	133	617	122	607
40.000004	108	534	94	541	88	600	91	558
31.748022	67	496	57	498	62	525	60	495
25.198421	47	433	36	417	41	452	37	564
20.000000	30	511	24	494	20	472	22	385
	180°		225°		270°		315°	
Resolution	fset	fset3	fset	fset3	fset	fset3	fset	fset3
96.000000	462	658	406	641	365	637	331	628
80.000008	339	640	311	620	282	579	240	624
63.496048	216	631	187	599	188	543	156	602
50.396847	139	598	122	573	116	508	113	570
40.000004	91	559	77	526	83	466	79	542
31.748022	57	475	42	455	58	397	59	516
25.198421	34	569	30	545	35	525	42	416
20.000000	21	365	19	379	23	321	31	451

Note: fset: the number of feature points used for continuous tracking; fset3: the number of feature points used for initializing tracking and recognizing images.

**Table 2:** Quantitative information about the reconstructed model's vertices, edges, faces, etc.

Properties					
Models	Quantities				
	Vertex	Edge	Face	Triangle	UV
Model 1	916230	2745256	1829026	1829026	946298
Model 2	102709	307339	204594	204594	107342
Model 3	862396	2583918	1721497	1721497	882512

**Table 3:** Effect video streaming frame rate.

Frame rate								
Scenes	Angles							
	0°	45°	90°	135°	180°	225°	270°	315°
Scenario 1	29.6	30.2	30.2	29.8	29.6	30.2	30.2	29.8
Scenario 2	30.2	30.2	29.9	29.7	30.3	29.8	29.8	29.9
Scenario 3	30.2	29.8	29.8	30.3	30.2	30.3	30.2	30.0

## Data Availability

The data used to support the findings of this study have been deposited in the DOI repository.
